The article "Standardised Mindfulness-Based Interventions in Healthcare: An Overview of Systematic Reviews and Meta-Analyses of RCTs" was retracted in 2019. Reasons: errors in the data; errors in the analysis; errors in the methods; errors in the results or conclusions.

# Standardised Mindfulness-Based Interventions in Healthcare: An Overview of Systematic Reviews and Meta-Analyses of RCTs

**DOI:** 10.1371/journal.pone.0124344

**Published:** 2015-04-16

**Authors:** Rinske A. Gotink, Paula Chu, Jan J. V. Busschbach, Herbert Benson, Gregory L. Fricchione, M. G. Myriam Hunink

**Affiliations:** 1 Department of Epidemiology, Erasmus MC, Rotterdam, the Netherlands; 2 Department of Psychiatry, section Medical Psychology and Psychotherapy, Erasmus MC, Rotterdam, the Netherlands; 3 Department of Radiology, Erasmus MC, Rotterdam, the Netherlands; 4 Department of Health Policy, Harvard University, Cambridge, United States of America; 5 Benson-Henry Institute for Mind Body Medicine, Massachusetts General Hospital, Harvard Medical School, Boston, United States of America; 6 Department of Psychiatry, Massachusetts General Hospital, Harvard Medical School, Boston, United States of America; 7 Department of Medicine, Massachusetts General Hospital, Harvard Medical School, Boston, United States of America; 8 Department of Health Policy and Management, Harvard School of Public Health, Boston, United States of America; Harvard Medical School, UNITED STATES

## Abstract

**Background:**

Mindfulness-based therapies are being used in a wide range of common chronic conditions in both treatment and prevention despite lack of consensus about their effectiveness in different patient categories.

**Objective:**

To systematically review the evidence of effectiveness MBSR and MBCT in different patient categories.

**Methods:**

A systematic review and meta-analysis of systematic reviews of RCTs, using the standardized MBSR or MBCT programs. We used PRISMA guidelines to assess the quality of the included reviews and performed a random effects meta-analysis with main outcome measure Cohen’s d. All types of participants were considered.

**Results:**

The search produced 187 reviews: 23 were included, covering 115 unique RCTs and 8,683 unique individuals with various conditions. Compared to wait list control and compared to treatment as usual, MBSR and MBCT significantly improved depressive symptoms (d=0.37; 95%CI 0.28 to 0.45, based on 5 reviews, N=2814), anxiety (d=0.49; 95%CI 0.37 to 0.61, based on 4 reviews, N=2525), stress (d=0.51; 95%CI 0.36 to 0.67, based on 2 reviews, N=1570), quality of life (d=0.39; 95%CI 0.08 to 0.70, based on 2 reviews, N=511) and physical functioning (d=0.27; 95%CI 0.12 to 0.42, based on 3 reviews, N=1015). Limitations include heterogeneity within patient categories, risk of publication bias and limited long-term follow-up in several studies.

**Conclusion:**

The evidence supports the use of MBSR and MBCT to alleviate symptoms, both mental and physical, in the adjunct treatment of cancer, cardiovascular disease, chronic pain, depression, anxiety disorders and in prevention in healthy adults and children.

The article "Standardised Mindfulness-Based Interventions in Healthcare: An Overview of Systematic Reviews and Meta-Analyses of RCTs" was retracted in 2019. Reasons: errors in the data; errors in the analysis; errors in the methods; errors in the results or conclusions.

## Introduction

Chronic illness is the largest cause of morbidity and mortality worldwide, causing 63% of all deaths[1]. Often there is no cure for these illnesses and patients face a high burden due to symptoms or side-effects of treatment. Consequently, stress, depression and anxiety are very common among these patients. Equally important as finding cures are efforts to provide chronic care and teach patients coping mechanisms to improve their quality of life. One adjunct therapy in chronic care that has gained popularity in the last 40 years is a secular variant of mindfulness.

Traditionally, mindfulness has been described as “a state of presence of mind which concerns a clear awareness of one's inner and outer experiences, including thoughts, sensations, emotions, actions or surroundings as they exist at any given moment” [2,3]. Unfortunately, such classical descriptions of mindfulness do not easily lend themselves to scientific investigation. Core components are usually described as follows: ‘full attention to internal and external experiences as they occur in the present moment’ and ‘an attitude characterized by non-judgment of, and openness to, this current experience’ [4–6]. Recently, Goyal et al. published a review of mindfulness interventions compared to active control and found significant improvements in depression and anxiety[7]. However, they included quite a heterogeneous group of meditation styles. Although the history of mindfulness as a way of life goes back 2500 years [2], a standardised version of mindfulness interventions for Western health care was only recently developed. In 1979, Jon Kabat-Zinn integrated mindfulness in his treatment of chronic pain patients and showed how changing the way patients relate to their pain can change their experience of pain [4]. His program, known as Mindfulness Based Stress Reduction (MBSR), spread quickly to other hospitals and other health problems. Teasdale, Williams and Segal converted MBSR to Mindfulness Based Cognitive Therapy (MBCT) for the treatment of depression. Since their initial promising results (50% relapse prevention in patients with 3 or more episodes of depression), studies repeatedly confirmed the benefit of MBCT in depression [8]. Subsequently, both MBSR and MBCT were well-defined and introduced in the care of various chronic conditions; MBSR, focusing more on the physical level of stress, found its way into supportive care for cancer, chronic pain, heart disease and fibromyalgia, whereas MBCT pays more attention to cognitive aspects and is used in the treatment of depression, anxiety, burn-out and eating disorders. Since mindfulness as a life style intervention is unlikely to have dangerous side-effects and can reduce stress, a risk factor for both mental and physical disorders, it is also being used in prevention (e.g. in education, parenting, the work place, pregnancy, and in prisons) [9], [10].

The article "Standardised Mindfulness-Based Interventions in Healthcare: An Overview of Systematic Reviews and Meta-Analyses of RCTs" was retracted in 2019. Reasons: errors in the data; errors in the analysis; errors in the methods; errors in the results or conclusions.

Despite the expanding application of MBSR and MBCT, the evidence for their use and the appropriate indications are debated. The aim of this study is to provide a systematic overview of the effectiveness of MBSR and MBCT in different patient populations in order to identify the patient categories in which these interventions are indicated.

## Methods

### Inclusion and exclusion criteria

We performed a systematic overview (based on Cochrane guidelines[11]) of systematic reviews of randomized controlled trials (RCTs) of the secular mindfulness techniques as Kabat-Zinn and Teasdale, Williams and Segal designed them (MBSR and MBCT, respectively). Although MBCT focuses more on cognitive skills, both MBSR and MBCT are delivered in an 8-week group course designed to cultivate the same non-judgmental, moment-to-moment awareness and involve the same meditative exercises and expectations for home practice, and were therefore judged to be equivalent in approach.

To be included the studies had to have the following characteristics: 1) be a systematic review of 2) randomized controlled trials with 3) MBCT and/or MBSR as the intervention 4) performed for treatment or prevention and 5) reporting any health outcome measure. Other types of mindfulness or meditation based techniques, such as Transcendental Meditation and Attention Control Training, were excluded. Also, articles that combined other types of interventions with MBSR or MBCT without calculating the effects separately for mindfulness were excluded. When reviews reported RCTs as well as other designs, they were only included if they reported the RCT results separately from the non-RCT studies. We also performed a separate search to check for RCTs published after the most recent systematic review. Unpublished dissertations and conference papers were excluded. As the aim of this study was to define indication areas, we did not restrict the search by patient population, publication date or number of RCTs reviewed.

### Search strategy

Six electronic databases were searched: PubMed, Embase, PsycInfo, Cochrane Reviews, Medline OvidSP and Web-of-Science. The databases were searched for English language publications using the following terms: “mindfulness” or “meditation” or “mindfulness-based stress reduction” or “MBSR” or “mindfulness-based cognitive therapy” or “MBCT”, in combination with “RCT” or “randomized” or “clinical trial” and “review” or “systematic” or “meta-analysis” (see for exact search strategy S1 Table).

The article "Standardised Mindfulness-Based Interventions in Healthcare: An Overview of Systematic Reviews and Meta-Analyses of RCTs" was retracted in 2019. Reasons: errors in the data; errors in the analysis; errors in the methods; errors in the results or conclusions.

### Study selection process

Reviews were independently selected by title and abstract by the first two authors. Any citation considered potentially relevant by at least one reviewer was retrieved in full text form in order to determine whether it met the selection criteria stated previously. Disagreements about the relevance of particular reviews were resolved by discussion with a third reviewer with methodological expertise. A log of rejected reviews along with reasons for their rejections is available in the supplementary material (S2 Table).

### Data extraction and quality assessment

The systematic reviews were evaluated independently by the first two authors for both content and quality. They extracted data based on the PRISMA guidelines for systematic reviews[12]. If information was missing or data were incomplete, the authors of the review were contacted or the RCTs concerned were retrieved in order to give an overview as thorough as possible. To assess the quality of the systematic reviews, a checklist was created using the validated PRISMA guidelines[12] (for items see Table 1).

**Table 1:** Quality assessment items based on the PRISMA criteria for systematic reviews.

Item	Question	Item on original checklist
1	Was the objective of the review explicitly described with reference to the participants, interventions, comparisons, and outcomes (PICO)?	PRISMA item 4
2	Were study eligibility criteria (inclusion/ exclusion criteria) and study selection process reported?	PRISMA item 6 + 9
3	Was a comprehensive literature search performed?	PRISMA item 7
4	Was the search strategy reported for at least one database?	PRISMA item 8
5	Was a list of studies (included and excluded) provided?	
6	Was study selection and data extraction done by at least two independent authors?	PRISMA item 10
7	Was the risk of bias of individual studies assessed and presented?	PRISMA item 12 + 19
8	Were also unpublished studies included (risk of publication bias)?	PRISMA items 15 + 22
9	If applicable, was the method for combining results appropriate?	PRISMA item 14 + 16
10	Were the strengths and limitations of the review addressed?	PRISMA item 25
11	Is the conclusion supported by the data, taking into account the quality of the studies?	PRISMA item 26
12	Were the findings interpreted independently of the funding source?	PRISMA item 27

### Main outcome measures and measures of effect size

Since we evaluated the effects of MBCT and MBSR in health care in general, we extracted both mental and physical outcome measures. We report the summarised RCT results of the reviews in different patient categories in order to address which indications are appropriate. No primary or secondary outcome measures in specific fields were pre-defined and all reported effect measures were considered.

The article "Standardised Mindfulness-Based Interventions in Healthcare: An Overview of Systematic Reviews and Meta-Analyses of RCTs" was retracted in 2019. Reasons: errors in the data; errors in the analysis; errors in the methods; errors in the results or conclusions.

### Data synthesis

Intergroup comparison effects (improvement intervention vs control group) are reported unless mentioned otherwise. If the intergroup results were insignificant, we also looked at intragroup differences in order to see if the intervention had at least a pre-post effect (which is already incorporated in significant intergroup effects). The control group includes: wait list control (WL), treatment as usual (TAU) or active treatment (AT). Results reported as a standardized mean difference (smd, including Cohen’s d and Hedges’ g) were combined using software specially designed for meta-analysis (RevMan version 5.3, 2014) [13]. The results are pooled by outcome (anxiety, depression, stress, quality of life and physical functioning), to indicate in which populations these symptoms are amenable to mindfulness. Data synthesis was performed with random effects analysis. Reviews that reported effect measures other than smd were excluded from the data synthesis due to incomparability (heterogeneity in effect measure). Since we included reviews instead of individual trials, there is a risk of multiple included RCTs. We therefore a priori set the maximum of double counting in the meta-analyses at 10% per patient category and excluded reviews that reported more duplicate data. Furthermore, in order to be totally transparent, in the supplementary material a table is provided to show exactly which RCTs were included more than once per meta-analysis (S3 Table).

## Results

### Study Selection

A total of 299 potentially eligible articles were identified, retrieved, and screened for potential inclusion (see for the flowchart the S1 Fig). 112 reviews were duplicate records. From the remaining 187 articles, 146 were excluded based on the abstract: 34 were not systematic reviews, 33 were not reviews of RCTs and 79 did not have MBCT or MBSR as intervention. Five results were conference abstracts and not yet published. The full text of the remaining 36 articles was reviewed. Eight articles were excluded because the RCT results were not reported separately and five were excluded due to too much overlap in RCTs with other reviews. All excluded articles and the reason for their rejection are listed in supplementary S2 Table. 23 reviews met our inclusion criteria and were reviewed by the first and second author. The search for RCTs published after the most recent included review gave 9 results, which are reported on at the end of the result section, together with 7 RCTs included in systematic reviews that were excluded from our review.

The article "Standardised Mindfulness-Based Interventions in Healthcare: An Overview of Systematic Reviews and Meta-Analyses of RCTs" was retracted in 2019. Reasons: errors in the data; errors in the analysis; errors in the methods; errors in the results or conclusions.

### Data extraction and quality assessment

Characteristics of the study, patient population, intervention, control condition, and outcome measures of the 23 included reviews are shown in Table 2.

**Table 2:** Study characteristics.

Author (year)	Design	Population (number of participants)	Intervention (number of RCT’s)	Control intervention	Outcome measure
Ledesma (2009)	Syst &Meta	Cancer (381)	MBSR (4)	2 TAU, 2 not specified	Mental health, physical health
Piet (2012)	Syst & Meta	Cancer (955)	Both (9)	6 WL, 3 TAU	Depression, anxiety
Cramer (2012)	Syst & Meta	Cancer (327)	MBSR (3)	TAU, 2 AT	Quality of life, mental health
Ott (2006)	Syst	Cancer (326)	MBSR (3)	WL, 2 AT	Mental health, sleep, nutrition
Smith (2005)	Syst	Cancer (268)	MBSR (3)	WL, TAU, AT	Mental health, sleep
Shennan (2011)	Syst	Cancer (215)	Both (3)	WL, 2 TAU	Anxiety, mood, mental health
Veehof (2011)	Syst & Meta	Chronic Pain (409)	MBSR (7)	3 WL, TAU, 3 AT	Mood, mental health
Cramer (2012)	Syst	Chronic Pain (117)	MBSR (3)	2 WL, AT	Pain intensity, disability, safety
Kozasa (2012)	Syst	Chronic Pain (208)	MBSR (2)	WL, TAU	Depression, quality of life
Abbott (2014)	Syst & Meta	Cardiovascular (557)	Both (9)	6 WL, TAU, 2 AT	Depression, anxiety, stress, hypertension
Bohlmeijer (2009)	Syst & Meta	Chronic somatic diseases (667)	MBSR (7)	WL	Mood, anxiety, mental health
Lakhan (2013)	Syst & Meta	Chronic somatic diseases (883)	Both (10)	6 WL, 4 AT	Symptom severity
Chiesa (2011)	Syst & Meta	Depression (781)	MBCT (14)	12 TAU, 2 AT	Depression (relapse), quality of life
Coelho (2007)	Syst	Depression (265)	MBCT (3)	TAU	Mood
Piet (2011)	Syst & Meta	Depression (593)	MBCT (6)	4 TAU, 2 AT	Depression relapse
Chen (2012)	Syst & Meta	Anxiety (1244)	Both (13)	8 WL, 5 AT	Anxiety
Klainin-Yobas (2012)	Syst & Meta	Mental disorders (964)	Both (13)	10 TAU, 3 AT	Mood, anxiety, mental health
Galante (2012)	Syst & Meta	Mental disorders (859)	MBCT (11)	10 TAU, AT	Depression (relapse), anxiety
Davis (2012)	Syst	Mental disorders (90)	Both (2)	WL, AT	Clinical functioning, mindfulness
Strauss (2014)	Syst & Meta	Mental disorders (550)	Both (11)	WL, 4 TAU, 6 AT	Anxiety, symptom severity
De Vibe (2012)	Syst & Meta	Mixed population (1942)	MBSR (31)	21 WL, 3 TAU, 7 AT	Mental health, physical health, quality of life, social function
Regehr (2012)	Syst & Meta	Healthy adults (247)	MBSR (5)	unknown	Mood, anxiety, stress
Burke (2009)	Syst	Children (330)	Both (2)	TAU, activities	Social skills, attention, temperament, stress

Syst = Systematic Review; Meta = Meta-analysis; MBSR = Mindfulness Based Stress Reduction; MBCT = Mindfulness Based Cognitive Therapy; TAU = treatment as usual; WL = waiting list; AT = Active Treatment

The results of the quality assessment are shown in Table 3. The inter-rater correlation was moderate (k = 0.48), and was influenced by structurally lower scoring of item 4 (search strategy reported) and item 9 (appropriate methods for combining results) by one reviewer due to different interpretation. The quality scores shown are those agreed upon after discussion. Nearly all reviews performed well on items related to the description of the objective, the literature search, and the study selection process (items 1–4). The list of included and excluded RCTs was not always complete (item 5). Although some reviews employed independent data extractors, many did not, and several were unclear about this item (item 6). Approximately half of the reviews assessed and presented the risk of bias of individual RCTs and the risk of publication bias (items 7 and 8). A meta-analysis of the individual RCTs was often not performed (item 9). In general, strengths and limitations were discussed, conclusions were supported by the data, and findings were interpreted independently of the funding source (items 10–12).

The article "Standardised Mindfulness-Based Interventions in Healthcare: An Overview of Systematic Reviews and Meta-Analyses of RCTs" was retracted in 2019. Reasons: errors in the data; errors in the analysis; errors in the methods; errors in the results or conclusions.

**Table 3:** Quality assessment of included reviews.

	Items	1	2	3	4	5	6	7	8	9	10	11	12
Ledesma		+	+	+	+	?	+	-	-	+	+	?	?
Piet (2012)		+	+	+	+	?	+	+	+	+	+	+	?
Cramer		+	+	+	+	?	+	+	?	N/A	+	+	+
Ott		?	?	?	+	?	?	-	+	N/A	?	?	?
Smith		+	+	+	+	?	+	-	+	N/A	?	+	?
Shennan		+	+	+	+	?	?	-	+	N/A	+	+	+
Veehof		+	+	+	+	?	?	+	+	+	+	+	?
Cramer		+	+	+	+	?	+	+	-	+	+	+	+
Kozasa		-	+	-	?	?	?	?	-	N/A	-	+	+
Abbott		+	+	+	+	-	+	+	?	+	+	+	+
Bohlmeijer		+	+	+	-	?	?	?	-	+	+	?	?
Lakhan		?	+	+	?	+	?	-	?	+	+	+	+
Chiesa		+	+	+	+	+	+	+	-	+	+	+	?
Coehlo		?	+	+	+	?	+	+	+	?	+	+	-
Piet (2011)		+	+	+	+	?	-	+	-	+	+	+	+
Chen		+	+	+	+	?	+	?	-	+	+	+	+
Klainin-Yobas		+	+	+	+	?	?	+	+	+	?	+	+
Galante		+	+	+	+	?	+	+	-	+	+	?	+
Davis		?	+	+	+	?	?	-	-	?	+	?	?
Strauss		+	+	+	+	-	?	+	+	+	+	+	+
De Vibe		+	+	+	-	+	+	+	+	+	+	+	+
Regehr		+	+	+	-	?	?	-	-	+	+	+	+
Burke		+	+	+	+	?	-	-	-	N/A	+	+	?

+ = yes;? = unclear;— = no; N/A = not applicable

### Synthesis of results

The results of the reviewed RCT’s are summarized below, categorized by patient population (see also Table 4). 115 unique RCTs were included, with a combined total of 8683 participants. 3830 individuals had various somatic conditions; 4276 patients had various psychological problems and the remaining 577 subjects were recruited from the general population. Effect sizes used were Cohen’s d, Hedges g, Standard Mean Difference, Weighted Mean Difference (wmd), T-value, Odds Ratio, Hazard Ratio and Risk Ratio. Of note, most systematic reviews demonstrated a significant effect size.

The article "Standardised Mindfulness-Based Interventions in Healthcare: An Overview of Systematic Reviews and Meta-Analyses of RCTs" was retracted in 2019. Reasons: errors in the data; errors in the analysis; errors in the methods; errors in the results or conclusions.

**Table 4:** Results.

Author (year)	Effect measure	Depression		Depression Relapse	Anxiety	Stress	Quality of Life	Pain	Mindfulness	Other
**Cancer**										
Ledesma (2009)	Cohen’s d									Mental health 0.37 (Physical health 0.17)
Piet (2012)	Hedges g	0.44			0.37				0.39	
Cramer (2012)	Smd	0.37			0.51					
Ott (2006)	T (paired sample test)	5.52			6.19	3.63				(Sleep); (nutrition)
Smith (2004)	Narrative	(Improved)								(Sleep)
Shennan (2011)	Narrative	Improved			Improved	Improved	(Improved)		Improved	
**Chronic Pain**										
Veehof (2011)	Smd	0.26			(0.55)		(0.25)	0.25		Physical health 0.43
Cramer (2012)	Narrative						WL, (AT)	WL, (AT)	(Improved)	(Self-efficacy)
Kozasa (2012)	Narrative	Improved					Improved			
**Cardiovascular disease**										
Abbott (2014)	Smd	0.35			0.50	0.38				Hypertension 0.78
**Chronic Somatic Diseases**										
Bohlmeijer (2009)	Hedges g	0.26			0.47	0.32				
Lakhan (2013)	Hedges g									Symptom severity MBSR 0.45; MBCT 0.64
**Depression**										
Chiesa (2011)	Wmd, OR	(11.24)		0.36 OR	13.8 bipolar, (2.34 soc ph)					
Coelho (2007)	HR			0.40–0.47						
Piet (2011)	RR	0.66								
**Anxiety**										
Chen (2012)	Smd				0.51					
**Mental Disorders**										
Klainin-Yobas (2012)	Cohen’s d	0.39	Improved		(CBT)					
Galante (2012)	Wmd, RR, smd	2.46 HAMD; 10.39 BDI	0.61 (RR)		0.42 (smd)					
Davis (2012)	Narrative	Improved			Improved	(AT)			Improved	Clinical functioning
Strauss (2014)	Hedges g									Symptom severity (0.75 MBSR), 0.39 MBCT
**Mixed Population**										
De Vibe (2012)	Hedges g	0.54			0.53	0.56	0.57		0.70	Mental health 0.53 Physical health 0.31
**Healthy adults**										
Regehr (2012)	Smd				0.73					
**Children**										
Burke (2009)	Cohen’s d				Improved	Improved				Attention 0.39–0.60 Mental health 0.28–0.92

Effect sizes reported as in reviews in different outcome measurements for the intergroup comparisons. Values are significant except when in parentheses. Smd = standard mean difference; OR = Odds Ratio; Wmd = weighted mean difference; HR = Hazard Ratio; RR = Risk Ratio. Interpretation: Cohen’s d, Hedges’g and smd: effect size 0–0.19 = no effect; 0.2–0.49 = small effect; 0.5–0.79 = medium effect; 0.8 and above = large effect. () = not significant. WL = compared to Wait list control; AT = compared to active treatment control

Also, 8 reviews were included in the meta-analysis based on reported intergroup smd’s of MBCT/MBSR and the pooled effect per outcome. Reviews that did not conduct a meta-analysis reporting in smd were excluded from our meta-analysis due to heterogeneity of effect size, but were only reviewed. The forest plots (Fig 1) demonstrate significant differences in favour of MBCT/MBSR. Three reviews that reported smd’s on our outcome measures were omitted from the meta-analyses which ensured that the number of double counted RCTs remained under 10% [14–16]. The meta-analysis on reviews with outcome depression had 3% double counting (1 out of 34 RCTs), anxiety 8.6% (3 out of 35 RCTs), both stress and quality of life had 0% double counting and physical functioning had 6% (1 out of 17 RCTs). An overview of the RCTs in each meta-analysis outcome and a more elaborate description of the results can be found in the online supplementary material (S3 Table).

The article "Standardised Mindfulness-Based Interventions in Healthcare: An Overview of Systematic Reviews and Meta-Analyses of RCTs" was retracted in 2019. Reasons: errors in the data; errors in the analysis; errors in the methods; errors in the results or conclusions.

**Fig 1:** Forest plots showing the effectiveness of mindfulness interventions compared with wait list control or treatment as usual on the outcomes a) Depression, b) Anxiety, c) Stress, d) Quality of life and e) Physical functioning in different populations. The size of the marker per review indicates the size of the study population. The breadth of the line indicates the 95%CI. All values lower than 0 indicate a significant difference in favour of MBSR/MBCT. Values between 0 and -0.2 indicate negligible effect; between -0.2 and -0.5 small effect; between -0.5 and -0.8 medium effect and lower than -0.8 a large effect.

### Mindfulness and Cancer

The search identified six systematic reviews covering 16 unique RCTs performed in 1668 unique cancer patients. 12 RCTs spread over two reviews were included in the meta-analysis, with one RCT duplication (8%). Most reviews found significant intergroup improvements in mental health but no significant results in physical health[16]. Significant improvements were demonstrated repeatedly in depressive symptoms, anxiety, stress, and quality of life [14,17–20]. Sleep quality did not change significantly; neither did body mass or fat consumption. A dose-response relationship was found between the number of minutes spent on meditating and improvement in total mood disturbance, and between the number of sessions attended and stress reduction [18], [20]. An association between the KIMS-subscale Observing [21] (a measure of mindfulness) and a decrease in anxiety, isolation and over-identification was also found.

### Mindfulness and Chronic Pain

For chronic pain patients we found three systematic reviews including 13 unique RCTs in 722 unique patients. One review containing 9 RCTs was included in the meta-analysis. Significant intergroup improvements were found in depressive symptoms, pain burden, and physical health, but neither in anxiety nor overall quality of life [22]. Pain intensity and pain disability decreased significantly and pain acceptance increased compared to wait list control but not when compared to a health education program. Self-efficacy showed no significant improvements. Quality of life favoured MBSR compared to the health education program but did not reach statistical significance when compared to wait list control [23]. MBSR also improved quality of life and depressive symptoms significantly in fibromyalgia patients [24].

The article "Standardised Mindfulness-Based Interventions in Healthcare: An Overview of Systematic Reviews and Meta-Analyses of RCTs" was retracted in 2019. Reasons: errors in the data; errors in the analysis; errors in the methods; errors in the results or conclusions.

### Mindfulness and cardiovascular disease

One review looked at the effects of MBSR and MBCT on psychological and physical outcomes in 577 cardiovascular patients in 9 RCTs [25]. Depression, anxiety and stress showed significant medium effects (smd 0.35 to 0.50), and hypertension improved with a significant smd of 0.78.

### Mindfulness and various chronic somatic diseases

Two reviews included 16 unique RCTs on MBSR and MBCT for various chronic somatic diseases (cancer, chronic pain, CVD, and fibromyalgia). In total 1331 unique patients were assessed. These reviews were excluded from the meta-analysis outcomes due to too much RCT overlap with other reviews in the meta-analysis. MBSR had a significant positive effect on depression symptoms, anxiety and psychological distress[26]. One of the reviews compared MBSR to MBCT for reducing symptom severity and found that MBCT was more effective, however no explanation was given[27].

### Mindfulness and Depression

Three systematic reviews of 17 unique RCTs with 1058 currently or recovered depressed patients were retrieved, none of which were included in the meta-analysis. The overall effect on depressive symptoms comparing MBCT with TAU was positive but not significant. However, in participants with 3 relapses or more, MBCT reduced depressive symptoms significantly between groups. Anxiety in bipolar patients was also reduced significantly[28]. The relapse rate decreased significantly in patients who had 3 depression episodes or more with a risk reduction of 43% compared to TAU[29]. Treatment in patients with 2 previous episodes, however, favoured TAU with a risk reduction of 49%. MBCT compared with antidepressants demonstrated a non-significant risk reduction of 20%[30].

### Mindfulness and anxiety

A review of 13 RCTs with a total of 1244 patients with different anxiety disorders found a significant beneficial effect on anxiety [31]. Interestingly, RCTs conducted in Western countries showed bigger effects than those conducted in Eastern countries.

### Mindfulness and various mental disorders

Four reviews assessed the effect of MBCT and MBSR among people with various mental disorders. 30 unique RCTs among 1974 unique participants were included. Two were included in the meta-analysis without overlap as one reported on depression [32], the other on anxiety[15]. Significant benefits were found in depressive symptoms, depression relapses and anxiety, and a significant increase in metacognitive awareness of negative thoughts and feelings was found. Relapse prevention was still significant at 1 year follow-up [15]. Not all RCTs, however, showed significant changes in relapse occurrence, and cognitive behavioural therapy was found to be superior to MBSR in reducing social anxiety [32]. In bipolar disorder, significant lower depression and anxiety scores were found. In schizophrenia there was significant intragroup improvement in clinical functioning and mindfulness of distressing thoughts and images; intergroup differences, however, did not reach significance [33]. In patients with a current anxiety or depression disorder, MBCT showed more effect than MBSR. Compared with WL and TAU there was a very large effect on symptom severity, however compared with active treatment this effect almost disappeared[34].

The article "Standardised Mindfulness-Based Interventions in Healthcare: An Overview of Systematic Reviews and Meta-Analyses of RCTs" was retracted in 2019. Reasons: errors in the data; errors in the analysis; errors in the methods; errors in the results or conclusions.

### Mindfulness in Mixed populations

We included one review with heterogeneous populations, as excluding it would result in missing 18 unique RCTs [35]. Compared to meditation alone, MBSR had a positive effect on perceived stress, rumination and forgiveness. Compared to muscle relaxation in a study population of 31 inmates, however, MBSR caused no substantial differences in anger, egocentricity, stress reactivity or salivary cortisol. Mindfulness combined with light therapy diminished skin clearing rates of psoriasis patients significantly. There was no significant effect in treatment outcomes in a study with drug addicts. In a neuroimaging study of healthy employees a MBSR intervention produced increases in left-sided anterior cortical activation, which is associated with positive affect, and significant increase in influenza antibody titres.

### Mindfulness in Healthy populations

Among healthy subjects, 5 RCT’s were performed in 247 students[36]. Anxiety decreased significantly compared to students that did not receive MBSR, and although depressive symptoms and stress also seemed to improve, this effect was analysed together with the effect of cognitive behavioural therapy, so the results could not be reported here.

### Mindfulness and Children

One review assessed the effects of mindfulness in 330 children studied in two RCTs. Significant intergroup improvements were reported in anxiety, teacher-rated attention, social skills and objective measures of selective (visual) attention, but not in sustained attention. A study with adolescents under current or recent psychiatric outpatient care showed significant intergroup improvements in stress, anxiety, and several psychopathological symptoms. The study also found that more time spent in sitting meditation predicted improved functioning and a decline in depression and anxiety symptoms. A study including non-clinical 4–5 year olds indicated significant improvements in executive functioning on teacher ratings, but not on parent ratings [37].

The article "Standardised Mindfulness-Based Interventions in Healthcare: An Overview of Systematic Reviews and Meta-Analyses of RCTs" was retracted in 2019. Reasons: errors in the data; errors in the analysis; errors in the methods; errors in the results or conclusions.

### Individual RCTs

Our search for individual RCTs not included in assessed systematic reviews resulted in 16 studies. Although some conclusions were not congruent with those in the reviews, overall the results supported use of the program. One RCT reports that currently non-depressed patients with one or two relapses benefit more from MBCT than patients with 3 or more relapses [38], whereas an included review [30] claimed the opposite. Note that both groups improved significantly in both studies, but results disagreed on which group improved more. Furthermore, the improvements in 39 Chinese chronic pain patients were not significant compared to active pain management [39] and no physical improvements were found in 86 elderly COPD patients [40].

Apart from these results, the other 13 RCTs demonstrated similar results as reported in the reviews: significant improvements in perceived stress, quality of life, symptom severity, anxiety and depression in patients with cancer [41], HIV [42], depression [43], mental disorders [44], ulcerative colitis [45], fibromyalgia [46], nonspecific chronic pain [47] [48], insomnia [49] and Parkinson [50], and in healthy participants [51–53].

## Discussion

### Summary of main results

This review provides an overview of more trials than ever before and the intervention effect has thus been evaluated across a broad spectrum of target conditions, most of which are common chronic conditions. Study settings in many countries across the globe contributed to the analysis, further serving to increase the generalizability of the evidence. Beneficial effects were mostly seen in mental health outcomes: depression, anxiety, stress and quality of life improved significantly after training in MBSR or MBCT. These effects were seen both in patients with medical conditions and those with psychological disorders, compared with many types of control interventions (WL, TAU or AT). Further evidence for effectiveness was provided by the observed dose-response relationship: an increase in total minutes of practice and class attendance led to a larger reduction of stress and mood complaints in four reviews [18,20,37,54].

### Strengths and limitations of the systematic review

As one of the aims was to identify how different patient populations respond to mindfulness, we included a heterogeneous group of populations. However, even when we categorized them by diagnosis, some reviews included very heterogeneous populations themselves. Excluding these would cause us to miss 18 unique RCTs, so we defined a category ‘mixed population’ representing heterogeneous patient populations. Although we tried to report their results as clearly as possible, interpretation of this group’s effects is difficult.

The article "Standardised Mindfulness-Based Interventions in Healthcare: An Overview of Systematic Reviews and Meta-Analyses of RCTs" was retracted in 2019. Reasons: errors in the data; errors in the analysis; errors in the methods; errors in the results or conclusions.

Also, though MBSR and MBCT were considered equal in approach, the small heterogeneity of interventions could have resulted in some bias towards the null, thereby strengthening the validity of our findings of consistent effects of these interventions. Due to the nature of the intervention, double blinding cannot be implemented in RCTs of mindfulness, leading to a risk of bias. As with all RCTs involving an unblinded treatment, patients’ attitudes towards mindfulness alone may lead to an effect: a placebo effect in the active intervention group and disappointment in the control group for not receiving mindfulness (“frustrebo response”)[55]. Whereas a placebo effect would overestimate the effect size, the frustrebo response can lead to control patients starting mindfulness on their own, underestimating the effect size. However, it might also be that frustration of not receiving the intervention leads to worse depression or anxiety scores in the control group, resulting in an overestimation of the effect. Because of the need for active participation, it is desirable that mindfulness is actively chosen: as bias is inherent in self-selected samples, the results might be extrapolated only to patients or participants who are interested in and able to participate in the intervention [16]. This, however, applies to most types of psychotherapy: motivation for and trust in the technique are essential. Furthermore, some RCTs were included in multiple reviews, so overlap in the described results exists. However, this was not believed to cause an overestimation of effect as the description of effect itself does not change by the number of RCTs. In the meta-analysis the overlap was 8% at most, reducing the overestimation inevitable in reviewing reviews to a minimum. There is risk of publication bias since we included only published reviews, although several of the included reviews contained both published and non-published RCTs. Also, despite our separate RCT search we may have missed RCTs by excluding reviews that analysed them together with other study designs or interventions (such as yoga). Although most individual RCTs included are in line with the results reported in the reviews, some did report disputing conclusions regarding Chinese patients treated for pain and elderly COPD patients.

The article "Standardised Mindfulness-Based Interventions in Healthcare: An Overview of Systematic Reviews and Meta-Analyses of RCTs" was retracted in 2019. Reasons: errors in the data; errors in the analysis; errors in the methods; errors in the results or conclusions.

Another limitation may be that the heterogeneity of studies within the systematic reviews may be masked within the overview, as each systematic review has a single confidence interval that may or may not contain all the point estimates of the studies in that review. This could give a false impression of homogeneity at the meta-meta level.

Several reviews reported that the quality of included RCTs corresponded with the effect sizes [31,32], with lower quality RCTs tending to report a larger effect than high-quality RCTs. Some were pilot studies presenting preliminary results without confirmatory evidence. Despite these limitations, the quality of the reviews was generally quite high and suggests that the conclusions drawn from these pragmatic RCTs provide relevant estimates of effectiveness in clinical practice. The interventions were compared repeatedly to both wait list and treatment as usual subjects. A recent review compared meditation to only active control groups, and although lower, also found a beneficial effect on depression, anxiety, stress and quality of life. This review was excluded in our study for its heterogeneity of interventions [7].

### Clinical implications

In chronic care, both MBCT and MBSR help patients cope with pain, depressive symptoms, anxiety, and stress, which improves their quality of life. In mental health, there are more ambiguous results: some disorders improve, others such as social anxiety and schizophrenia respond better to traditional treatment. In prevention, mindfulness is valuable in reducing stress and other psychopathological symptoms that might otherwise develop into clinical conditions. In education and parenting, teaching children how to cope with stress and upsetting situations in a mindful way can help them deal with those aspects of life in the future. We also have to take into account the meaning of effect sizes in different populations: an effect size of 0.5 in anxiety might mean something different in anxiety patients than in cancer patients. In the first case, depending on the exact anxiety disorder, other treatments might have a larger effect. In cancer patients however, reducing this much anxiety may have a huge impact on quality of life. This discrepancy helps make a distinction as to where to apply mindfulness as adjunct treatment.

There are several benefits of adding mindfulness to usual treatment. First, MBSR and MBCT are easy to implement and they allow patients to take a more active role in their treatment. Second, there is little emotional and physical risk involved. Third, the costs are relatively low as one trainer can lead a rather large group and most exercises can be done at home, without the help of external means [17]. However, they do require commitment in both adherence and time of both the patient and the therapist.

The article "Standardised Mindfulness-Based Interventions in Healthcare: An Overview of Systematic Reviews and Meta-Analyses of RCTs" was retracted in 2019. Reasons: errors in the data; errors in the analysis; errors in the methods; errors in the results or conclusions.

### Gaps in evidence

Aim of this review was to assess in which populations MBSR and MBCT are effective, and in which not. Most insignificant effects found were based on pilot studies using outcome measures that are only indirectly affected by mindfulness (e.g. nutrition, HIV, psoriasis, drug addiction), therefore no definitive conclusions can be drawn for these outcome measures.

Since MBSR and MBCT consist of not just meditation, but also psycho-education and yoga-like exercises, it is difficult to pinpoint which aspect contributes most to the observed improvements. According to psychological theory [56], stress is usually caused by an external factor which evokes fear, anger, or other states of discontentment. Stress is also experienced proportionately; the larger the discrepancy between the actual and desired situation, the higher the level of stress. Apart from the initiating event, individuals themselves tend to magnify stress by worrying about the cause and consequences of the event, which often evokes more stress than the event alone. Mindfulness intervenes in this psychological process by creating a different relationship with both the event and the internal response to the event. Chronic as opposed to acute conditions respond particularly well to mindfulness techniques since acceptance and reflection may be more applicable to chronic symptoms than to acute symptoms. In acute settings the undesired situation may still be altered, making acceptance untimely.

Support for this theory of stress reduction by coping with psychological stress factors is found in the demonstrated physiological effects of mindfulness. Blood pressure, heart rate, respiration rate and oxygen consumption have been shown to respond favourably to mindfulness [57,58]. Similar physiological effects are seen in the relaxation response [59], [60]. It activates the autonomic nervous system to release endorphins and serotonin, and the parasympathetic response influencing endocrine and immune responses [61].

### Future research

Future research will benefit from creative strategies that measure placebo effects and non-specific effects, and distinguish these from actual effects. Nevertheless, the reviews included in our overview are methodologically strong and demonstrate that MBSR and MBCT are effective for certain conditions. Since the available evidence demonstrates that mindfulness exceeds WL control, future research should probably focus on comparison with active treatment. Further research should also look more into the mechanisms whereby these therapies are efficacious. Alongside investigating working mechanisms, studies should also explore the cost-effectiveness of these interventions: as there are few if any side effects and there seem to be benefits for chronic patients, insight in financial consequences is useful for further practical implementation in health care.

The article "Standardised Mindfulness-Based Interventions in Healthcare: An Overview of Systematic Reviews and Meta-Analyses of RCTs" was retracted in 2019. Reasons: errors in the data; errors in the analysis; errors in the methods; errors in the results or conclusions.

## Conclusions

Although there is continued scepticism in the medical world towards MBSR and MBCT, the evidence indicates that MBSR and MBCT are associated with improvements in depressive symptoms, anxiety, stress, quality of life, and selected physical outcomes in the adjunct treatment of cancer, cardiovascular disease, chronic pain, chronic somatic diseases, depression, anxiety disorders, other mental disorders and in prevention in healthy adults and children.

## Supporting Information

S1 Fig Flow chart. (DOCX)

S1 Table Search strategy. (DOCX)

S2 Table Excluded articles and reason for exclusion (DOCX)

S3 Table Assessment of double counting per meta-analysis (DOCX)

S1 Text Extensive description of results categorized by patient population. (DOCX)
